The article "Role of miR-584-5p in Lipopolysaccharide-Stimulated Human Bronchial Epithelial Cell Inflammation and Apoptosis" was retracted in 2023. Reasons: signs of a paper mill; compromised peer review; unreliable results or conclusions.

# Role of miR-584-5p in Lipopolysaccharide-Stimulated Human Bronchial Epithelial Cell Inflammation and Apoptosis

**DOI:** 10.1155/2022/2408682

**Published:** 2022-04-11

**Authors:** Bo Zhang, Qing Zhang, Linying Yang, Hongfei Zheng, Guifen Pang, Mingzhen Zhao, Bo Sun, Jie Cao

**Affiliations:** ^1^Department of Respiratory and Critical Care Medicine, Tianjin Medical University General Hospital, Tianjin 300052, China; ^2^Department of Respiratory and Critical Care Medicine, Affiliated Hospital of Chengde Medical College, Chengde 067000, Hebei, China

## Abstract

Acute lung injury (ALI)/acute respiratory distress syndrome is a common clinical syndrome characterized by respiratory failure. MicroRNAs (miRNAs) are closely related to ALI and acute respiratory distress syndrome. TargetScan software analysis showed that miR-584-5p can bind to the 3ʹ noncoding region of *TLR4*, which is involved in the occurrence and development of ALI, thereby affecting the inflammatory pathway and inflammation development. Thus, we aimed to determine whether miR-584-5p affects ALI. Human bronchial epithelial (16-HBE) cells were transfected with miR-584-5p mimics or inhibitors and then stimulated with lipopolysaccharide (LPS).The cell viability, apoptosis, release of proinflammatory factors, mTOR, and NF-*κ*B pathway protein expression were evaluated respectively. Mimic584 increased, whereas inhibitor584 decreased, LPS-stimulated inflammation. The protein expression of inflammatory factors was significantly increased in 16-HBE cells in the mimic584 + LPS group and decreased in the inhibitor584 + LPS group. Mimic584 activated mTOR and the NF-*κ*B-related proteins P65 and p-p65, whereas inhibitor584 inactivated the proteins in 16-HBE cells. Overexpression of miR-584 significantly promoted apoptosis in LPS-stimulated 16-HBE cells. There were no differences in the proliferation and cell cycle of LPS-stimulated 16-HBE cells regardless of mimic584 or inhibitor584 transfection. Collectively, we demonstrated that inhibitor584 can alleviate ALI-induced expression of inflammatory factors via mTOR signaling and the NF-*κ*B pathway. In conclusion, we found that inhibitor584 transfection could be a potential therapeutic strategy for ALI.

## 1. Introduction

Acute lung injury (ALI)/acute respiratory distress syndrome, a common clinical syndrome, refers to an acute, diffuse lung injury and the development of acute respiratory failure caused by various intrapulmonary and extrapulmonary pathogenic factors, resulting in the inflammation and apoptosis of alveolar epithelial cells [1]. MicroRNAs (miRNAs) are a class of endogenous, noncoding small RNA molecules that are 19–23 nucleotides in length [2]. miRNAs are important gene regulatory factors with partial complementary sites to untranslated regions of target mRNAs to repress the translation or cause the degradation of these mRNAs [3]. miRNAs play a major role in the progression of ALI and acute respiratory distress syndrome [4]. TargetScan (http://www.targetscan.org/) has been employed to predict the target genes of miR-584-5p; miR-584 can bind to the 3ʹ noncoding region of TLR4, thereby affecting the inflammatory pathway and inflammation development. To date, the effect of miR-584 on ALI and acute respiratory distress syndrome has been poorly understood, and most previous studies on miR-584 are related to tumors. The overexpression of miR-584 inhibits cell viability, migration, and proliferation and increases apoptosis in different carcinomas [5–11].

Hu et al. [12] demonstrated that mTOR plays an important role in lipopolysaccharide (LPS)-induced ALI in vivo. A bioinformatic analysis indicated *MIS12* as the target gene of miR-584-5p. In this study, the effect and mechanism of action of miR-584-5p on the inflammatory response of LPS-induced ALI were explored. In particular, a novel mechanism was investigated to identify potential targets for the treatment of ALI and biological indicators to determine the prognosis of ALI. For this purpose, human bronchial epithelial (16-HBE) cells were transfected with miR-584 mimics or inhibitors and then incubated with LPS. Next, we evaluated cell viability, apoptosis, proinflammatory factor release, mTOR expression, and the expression of proteins in the NF-*κ*B pathway to elucidate the role of miR-584-5p in LPS-stimulated 16-HBE cells.

## 2. Materials and Methods

### 2.1. Cell Culture

16-HBE cell line was obtained from the Basic Department of Chengde Medical College (Chengde, China). The cells were cultured in RPMI-1640 medium supplemented with 10% fetal bovine serum (Vivacell, Shanghai, China) and 1% penicillin/streptomycin (Invitrogen, Carlsbad, CA, USA) in a humidified 37 °C incubator with 5% CO_2_ [13]. The cells (approximately 4 × 10^5^/well) were plated in six-well plates and incubated for 24 h [14].

### 2.2. Cell Transfection

To achieve miR-584-5p overexpression or silencing in 16-HBE cells, mimic negative control (mimicNC), mimic miR-584 (mimic584), inhibitor negative control (inhibitorNC), and inhibitor miR-584 (inhibitor584) were purchased from Zhongshi Gene Technology Co., Ltd. (Tianjin, China) (Tables 1 and 2) and transfected into 16-HBE cells using Lipofectamine 3000 (Invitrogen, USA) according to the manufacturer's instructions. After 24 h of transfection, the cells were incubated with LPS (100 µg/mL; Sigma, St. Louis, MO, USA) for 24 h.

### 2.3. RNA Extraction and qRT-PCR

The total RNA was extracted from 16-HBE cells using the Superbrilliant 6 min high-purity RNA extraction kit (Tianjin, China) according to the manufacturer's instructions and was reverse-transcribed to cDNA using a FastKing RT Reagent (Tiangen, China). qRT-PCR was performed using an automatic fluorescent PCR analyzer (Roche Molecular Systems, Branchburg, NJ, USA) with SYBR Green SuperReal PreMix Plus and the following primers (Rockville, MD, USA): interleukin-1 (*IL-1*) forward, 5ʹ-TGTATGTGACTGCCCAAGATGAAG-3ʹ and reverse, 5ʹ-AGAGGAGGTTGGTCTCACTACC-3ʹ; interleukin-6 (IL-6) forward, 5ʹ- AGACAGCCACTCACCTCTTCAG-3ʹ and reverse, 5ʹ- TTCTGCCAGTGCCTCTTTGCTG-3ʹ; interleukin-8 (IL-8) forward, 5ʹ-GAGAGTGATTGAGAGTGGACCAC-3ʹ and reverse, 5ʹ- CACAACCCTCTGCACCCAGTTT-3ʹ; tumor necrosis factor-*α* (TNF-*α*) forward, 5ʹ-CTCTTCTGCCTGCTGCACTTTG-3ʹ and reverse, 5ʹ-ATGGGCTACAGGCTTGTCACTC-3ʹ; macrophage inflammatory protein-1*α* (MIP-1*α*) forward, 5ʹ-ACTTTGAGACGAGCAGCCAGTG-3′ and reverse, 5ʹ- TTTCTGGACCCACTCCTCACTG-3′; monocyte chemoattractant protein-1 (MCP-1) forward, 5ʹ-AGAATCACCAGCAGCAAGTGTCC-3ʹ and reverse, 5ʹ-TCCTGAACCCACTTCTGCTTGG-3ʹ.

After LPS stimulation, the total RNA was extracted from 16-HBE cells using the Superbrilliant Cell miRNA Extraction Kit (Tiangen, China) according to the manufacturer's protocol. The miRNA expression was analyzed using a miRNA reverse transcription reagent (Tianjin, China). qRT-PCR was performed using the automatic fluorescent PCR analyzer (Roche Molecular Systems, Mannheim, Germany) with the Supersmart TaqMan miRNA Quantitative PCR Probe (Tianjin, China) for miR-584-5p and RNU6 (internal group). The expression of miRNAs and mRNAs was normalized to that of U6 and GAPDH using the 2-ΔΔCt method, respectively.

### 2.4. Western Blotting

The cells were lysed in a lysis buffer containing protease inhibitors (50 mM Tris-HCl (pH 8), 50 mM NaCl, and 0.5% NP-40) [15]. Equal amounts of proteins were separated using sodium dodecyl sulphate-polyacrylamide gel electrophoresis and transferred on to polyvinylidene fluoride membranes. After blocking with 5% nonfat milk, the membranes were immunoblotted with primary antibodies against IL-1, IL-6, IL-8, TNF-*α*, MIP-1*α*, MCP-1, Bax, Bcl-2, cleaved caspase 3, cleaved caspase 12, p65, p-p65, mTOR, and GAPDH at a dilution of 1 : 1000 and incubated overnight at 4 °C. The membranes were then washed with Tris-buffered saline with Tween-20, exposed to horseradish peroxidase-conjugated goat anti-rabbit secondary antibodies (1 : 5000; Santa Cruz, USA), and analyzed using an ECL detection system (ApplyGen, Beijing, China).

### 2.5. Cell Viability Assay

Cell viability was assessed using the Cell Counting Kit-8 (CCK-8) and Proliferation Detection Kit (ReportBio, Hebei, China). Briefly, approximately, 4 × 10^4^ cells were seeded in 96-well plates, transfected with miR-584-5p mimics or inhibitors, stimulated with LPS, treated with 20 *μ*L of CCK-8 solution, and cultured for 1 h. The absorbance of the reaction system was measured spectrophotometrically at 450 nm [16] (Thermo Fisher Scientific, Shanghai, China).

### 2.6. Flow Cytometric Analysis of Cell Cycle and Apoptosis

Cell cycle and apoptosis were analyzed using flow cytometry. After transfection and LPS stimulation, the cells were digested with trypsin and centrifuged at 300 × g for 5 min. Before flow cytometric detection, the cells were washed carefully with phosphate-buffered saline (twice), fixed with 75% ethanol before storage at −20 °C overnight, and stained with propidium iodide solution (500 *μ*L) for 15 min at 30 °C for cell cycle analysis [17]. Apoptosis was determined by staining with Annexin V and PI (BD Biosciences, Franklin Lakes, NJ). Briefly, 16-HBE cells were incubated at a density of 4 × 10^5^/well in a six-well plate with the corresponding treatments. The cells were then washed with ice-cold PBS twice after digesting with trypsin, centrifuged at 800 g for 5 min, stained with 5 *μ*L of Annexin V and 5 *μ*L of PI, and incubated with 100 *μ*L of binding buffer for 15 min at 30 °C in the dark. The fluorescent signal was further analyzed using flow cytometry after the reaction volume was made up to 500 *μ*L by adding binding buffer. Data were acquired using a FACScan flow cytometer (BD Biosciences, Franklin Lakes, NJ, USA).

### 2.7. Statistical Analysis

Data are presented as mean ± standard deviation. Analysis of variance was used to compare the data with Social Sciences (SPSS) software version 26.0. The least significant difference (LSD) method was used to compare indexes between groups. Statistical significance was set at *P* < 0.05.

## 3. Results

### 3.1. MIS12 Is a Target Gene of miR-584-5p

To identify the target genes of miR-584, the TargetScan database [18] was used. miR-584-5p was found to regulate the expression of approximately 1000 genes. In particular, TargetScan predicts that *MIS12* is a putative target gene of miR-584-5p. The alignment of miR-584 and MIS12 is detailed in Figure 1(a). Next, the transfection efficiency was determined using Western blotting [19]. The results showed that the miR-584-5p level significantly changed after transfection. Western blotting revealed that the miR-584 expression resulted in a decrease in the MIS12 level; however, the MIS12 level was considerably enhanced in inhibitor584-transfected cells compared with that in normal and mimic584-transfected cells (Figure 1(b)).

Mimic584 increased and inhibitor584 decreased LPS-induced inflammation in 16-HBE cells.

We examined how miR-584-5p regulates the gene expression in HBE cells using qRT-PCR and Western blotting. To verify the effect of miR-584 on the inflammatory response induced by LPS, 16-HBE cells were transfected with mimicNC, mimic584, inhibitorNC, and inhibitor584 for 24 h and stimulated with LPS for 24 h. The total RNA was extracted from the cells to detect RNA and protein expression. The qRT-PCR results revealed that mimic584 + LPS-treated cells showed a significant increase in IL-1, IL-6, IL-8, TNF-*α*, MCP-1, and MIP-1*α* mRNA expression compared with mimicNC- and mimicNC + LPS-treated cells (Figure 2(a)). IL-8 expression was considerably reduced in inhibitor584 + LPS-treated 16-HBE cells compared with that in inhibitorNC-, inhibitor584-, and inhibitorNC + LPS-treated cells (Figure 2(b)). In general, these results showed that miR-584-5p overexpression increased the expression of inflammatory factors and chemokines, and the IL-8 mRNA expression was significantly attenuated by inhibitor584 transfection.

The TNF-*α* protein expression was significantly higher in mimic584 + LPS-treated cells than in mimicNC-, mimicNC + LPS-, and mimic584-treated cells; IL-1 protein expression was significantly higher in mimic584 + LPS-treated cells than in mimicNC-treated cells; and IL-6, IL-8, and MIP-1*α* protein expressions was significantly lower in mimicNC-treated cells than in mimic584-, mimicNC + LPS-, and mimic584 + LPS-treated cells. However, IL-6, TNF-*α*, and MIP-1*α* protein expression was considerably attenuated in inhibitor584 + LPS-treated cells compared with that in inhibitorNC-, inhibitorNC + LPS-, and inhibitor584-treated cells; the IL-8 protein expression was considerably attenuated in inhibitor584-transfected cells compared with that in inhibitorNC- and inhibitorNC + LPS-treated cells (Figure 3).

### 3.2. Apoptosis in LPS-Stimulated HBE Cells Transfected with mimic584 or inhibitor584

We assessed the expression of apoptotic indicators in all HBE cell groups. The expression of the proapoptotic proteins Bax, cleaved caspase 3, and cleaved caspase 12 was significantly higher in mimic584 + LPS-treated cells than in mimicNC-, mimic584-, and mimicNC + LPS-treated cells. The level of antiapoptotic protein Bcl-2 was significantly attenuated in mimic584 + LPS-treated cells compared with that in mimicNC + LPS-treated cells. In contrast, the caspase 12 expression was considerably attenuated in inhibitor584-transfected cells compared with that in inhibitorNC- and inhibitorNC + LPS-treated cells. The level of antiapoptotic protein Bcl-2 was significantly higher in inhibitor584 + LPS-treated cells than in inhibitorNC-treated cells (Figure 4).

Mimic584 activated and inhibitor584 inactivated mTOR and the NF-*κ*B-related proteins P65 and p-p65 in HBE cells.

The NF-*κ*B pathway is involved in the regulation of inflammatory responses [20]. Thus, we examined the involvement of mTOR and the NF-*κ*B-related proteins P65 and p-p65 in ALI in HBE cells in vitro. The expression of p-p65 and mTOR gradually increased in mimic584 + LPS-treated cells and decreased in inhibitor584 + LPS-treated 16-HBE cells (Figure 5). Collectively, miR-584-5p regulated LPS-induced cell injury via mTOR signaling and the NF-*κ*B pathway; mTOR activated the NF-*κ*B pathway and promoted HBE cell damage.

### 3.3. Effects of miR-584-5p on 16-HBE Cell Proliferation

The CCK-8 assay revealed that there was no difference in the proliferation of LPS-stimulated 16-HBE cells regardless of mimic584 or inhibitor584 transfection (*P* > 0.01; Figure 6).

### 3.4. Cell Cycle Analysis Using Flow Cytometry

The relevance of cell cycle interruption was analyzed using flow cytometry, which indicated that miR-584-5p mimics and inhibitors did not cause cell cycle arrest at any phase (G1/G2/S; Figure 7).

### 3.5. Overexpression of miR-584 Associated with Apoptosis

Cell apoptosis analysis using flow cytometry revealed a significant (*P* < 0.05) increase in the apoptosis rate in the mimic584 + LPS cells than in mimicNC, mimic584, and mimicNC + LPS cells. However, inhibitor584 + LPS treatment led to opposite results, with a considerably reduced apoptosis rate (Figure 8). This suggests that the absence of miR-584 sensitized cells to inhibit LPS-induced apoptosis. Conclusively, these results indicate that inhibitor584 plays an important role in inhibiting LPS-induced apoptosis (Figure 8).

## 4. Discussion

The current study demonstrated that mimic584 can activate inflammatory responses in bronchial epithelial cells, whereas inhibitor584 can inactivate them. The mechanism of activation of miR-584-5p was via mTOR signaling and the NF-*κ*B pathway. In addition, the levels of proinflammatory cytokines stimulated by LPS correlated with the miR-584-5p level.

ALI is a pathophysiological process involving bronchial epithelial cells, endothelial cells, and inflammatory cells [21]. Thus, in this study, we examined the effect of miR-584-5p on ALI-induced bronchial epithelial cell injury. miR-584 regulated the expression of a number of proinflammatory factors in bronchial epithelial cells in vitro, and this is contrary to the findings reported by Zhang et al. [22]. Furthermore, a bioinformatic analysis [23] demonstrated that miR-584-5p targets the *TLR4* expression, thereby enhancing the inflammatory response of bronchial epithelial cells [24]. Here, inhibitor584 reduced inflammation by inhibiting the release of inflammatory cytokines. Subsequently, we demonstrated that miR-584-5p, which was abundant in mimic-584 + LPS-treated 16-HBE cells, increased the expression of inflammatory and proinflammatory factors associated with ALI via mTOR signaling and the NF-*κ*B pathway. Moreover, mimic-584-transfected 16-HBE cells presented increased gene expression of relevant cytokines. In contrast, inhibitor584 transfection improved LPS-induced lung injury by decreasing mTOR and NF-*κ*B protein expression. Our experiment confirmed for the first time that overexpressing miR-584 promotes inflammation in bronchial epithelial cells and silencing miR-584 decreases inflammation during ALI.

Several studies have indicated that autophagy and the NF-*κ*B pathway play important roles in different animal and cell models of ALI [25, 26]. Studies [27, 28] have also revealed that viral infections, such as H5N1 infection, can cause lung epithelial cell autophagy and NF-*κ*B activation. Preventing autophagy can not only inhibit epithelial cell death but also improve H5N1-induced ALI. Here, we found that the activation of mTOR and the NF-*κ*B signaling pathway increased the expression of inflammatory factors [29] IL-1, IL-6, IL-8, TNF-*α*, MCP-1, and MIP-1*α*. Thus, inhibitor584 may exert its therapeutic potential, that is, decreasing inflammatory factor expression, through the inactivation of mTOR and the NF-*κ*B pathway.

This study had some limitations. The efficacy of miR-584 in an animal model was not examined and bronchial epithelial cells may not actually reflect the genotype of alveolar epithelial cells. However, HBE cells are commonly used as surrogates for alveolar epithelial cells owing to the difficulty in storing and isolating lung epithelial cells.

## 5. Conclusions

Taken together, the results showed that silencing miR-584 effectively reduced the expression of inflammatory factors and that it may be an effective target for ALI treatment. It is possible that the protective effects may be due to other components and not only due to inhibitor584; therefore, further investigation is warranted.

We demonstrated that inhibitor584 had a beneficial effect on LPS-induced ALI via mTOR signaling and the NF-*κ*B pathway. Furthermore, we identified a novel mechanism through which inhibitor584 reversed bronchial epithelial cell injury.

## Figures and Tables

**Figure 1:** miR-584-5p directly targeted the expression of MIS12. (a) Complementary base pairing between miR-584-5p and *MIS12* was predicted using TargetScan. (b) 16-HBE cells were transfected with mimic negative control (mimicNC), mimic miR-584-5p (mimic584), inhibitor negative control (inhibitorNC), or inhibitor miR-584-5p(inhibitor584) for 24 h. MIS12 expression was measured using western blotting.  ^*∗*^*p* < 0.05 compared with the control, mimic584, and inhibitorNC groups. The experiments were performed at least three times independently. Data are presented as mean ± standard deviation (SD).

**Figure 2:** Effects of miR-584-5p on lipopolysaccharide (LPS)-stimulated 16-HBE cell injury. (a) 16-HBE cells were transfected with mimic negative control (mimicNC), mimic miR-584-5p (mimic584), inhibitor negative control (inhibitorNC), or inhibitor miR-584-5p (inhibitor584) for 24 h and then stimulated with LPS (100 µg/mL) for 24 h. The mRNA expression of *IL-1*, *IL-6*, *IL-8*, *TNF-α*, *MCP-1*, and *MIP-1α* in 16-HBE cells was measured using qRT-PCR. *GAPDH* served as an internal control.  ^*∗*^*p* < 0.05 compared with the mimicNC, mimicNC + LPS, and mimic584 groups; #*p* < 0.05 compared with the mimicNC and mimic584 groups. (b) ^*∗*^*p* < 0.05 compared with the inhibitorNC, inhibitor584, and inhibitorNC + LPS groups. The experiments were performed at least three times independently. Data are presented as mean ± standard deviation (SD).

**Figure 3:** Effect of miR-584-5p on inflammation in lipopolysaccharide (LPS)-stimulated 16-HBE cells. 16-HBE cells were transfected with mimic negative control (mimicNC), mimic miR-584-5p (mimic584), inhibitor negative control (inhibitorNC), or inhibitor miR-584-5p (inhibitor584) for 24 h and then treated with LPS (100 µg/mL) for 24 h. The expression of IL-1, IL-6, IL-8, TNF-*α*, MCP-1, and MIP-1*α* in the transfected 16-HBE cells was measured using western blotting.  ^*∗*^*p* < 0.05 compared with the mimicNC group; #*p* < 0.05 compared with the mimic584, mimicNC + LPS, and mimic 584 + LPS groups; △*p* < 0.05 compared with the mimicNC, mimic584, and mimicNC + LPS groups; ▲*p* < 0.05 compared with the mimicNC and mimic584 groups.  ^*∗*^*p* < 0.05 compared with the inhibitorNC, inhibitor584, and inhibitorNC + LPS groups; #*p* < 0.05 compared with the inhibitorNC, inhibitorNC + LPS, and inhibitor584 + LPS groups; △*p* < 0.05 compared with the inhibitorNC and inhibitor584 groups; ▲*p* < 0.05 compared with the inhibitor584, inhibitorNC + LPS, and inhibitor584 + LPS groups. The experiments were performed at least three times independently. Data are presented as mean ± standard deviation (SD).

**Figure 4:** Effect of miR-584-5p on apoptosis of lipopolysaccharide (LPS)-stimulated 16-HBE cells. 16-HBE cells were divided into eight groups: mimic negative control (mimicNC), mimic miR-584-5p (mimic584), mimic negative control + LPS (mimicNC + LPS), miR-584-5p mimic + LPS (mimic584 + LPS), inhibitor negative control (inhibitorNC), inhibitor miR-584-5p (inhibitor584), inhibitor negative control + LPS (inhibitorNC + LPS), and inhibitor miR-584-5p + LPS (inhibitor584 + LPS). 16-HBE cells in the mimicNC and mimicNC + LPS groups were transfected with mimic negative control (mimicNC); mimic584 and mimic584 + LPS groups were transfected with mimic miR-584-5p (mimic584); inhibitorNC and inhibitorNC + LPS groups were transfected with inhibitor negative control (inhibitorNC); and inhibitor584 and inhibitor584 + LPS groups were transfected with inhibitor miR-584-5p (inhibitor584). Apoptosis in the mimicNC-, mimic584-, inhibitorNC-, and inhibitor584-transfected 16-HBE cells after LPS treatment was evaluated using western blotting. The protein expression of GAPDH, Bax, Bcl-2, cleaved caspase 3, and cleaved caspase 12 in all groups was measured using western blotting.  ^*∗*^*p* < 0.05 compared with the mimicNC, mimic584, and mimicNC + LPS groups; #*p* < 0.05 compared with the mimic584 and mimicNC + LPS groups; △*p* < 0.05 compared with the mimicNC, mimicNC + LPS, and mimic584 + LPS groups.  ^*∗*^*p* < 0.05 compared with the inhibitor584, inhibitorNC + LPS, and inhibitor584 + LPS groups; ^#^*p* < 0.05 compared with the inhibitorNC group; △ *p* < 0.05 compared with the inhibitorNC and inhibitor584 groups; ^▲^*p* < 0.05 compared with the inhibitorNC and inhibitorNC + LPS groups. The experiments were performed at least three times independently. Data are presented as mean ± standard deviation (SD).

**Figure 5:** miR-584-5p regulated mTOR and the NF-*κ*B signaling pathway in lipopolysaccharide (LPS)-stimulated HBE cells. Representative western blot of mTOR, p65, and p-p65 expression in mimicNC-, mimic584-, inhibitorNC-, and inhibitor584-transfected HBE cells after LPS treatment. The expression of GAPDH, p65, p-p65, and mTOR was analyzed using western blotting.  ^*∗*^*p* < 0.05 compared with the mimicNC and mimic584 groups; #*p* < 0.05 compared with the mimicNC, mimic584, and mimicNC + LPS groups.  ^*∗*^*p* < 0.05 compared with the inhibitorNC, inhibitor584, and inhibitorNC + LPS groups; #*p* < 0.05 compared with the inhibitor584, inhibitorNC + LPS, and inhibitor584 + LPS groups. The experiments were performed at least three times independently. Data are presented as mean ± standard deviation (SD).

**Figure 6:** Viability of transfected HBE cells. (a) and (b) Viability of mimicNC-, mimic584-, inhibitorNC-, and inhibitor584-transfected 16-HBE cells after lipopolysaccharide (LPS) treatment was analyzed using the Cell Counting Kit-8(CCK-8) assay. The experiments were performed at least three times independently. Data are presented as mean ± standard deviation (SD).

**Figure 7:** Effects of miR-584-5p on the cell cycle of 16-HBE cells. After treatment with 75% glacial ethanol, 16-HBE cells were stained with propidium iodide solution (500 *μ*L) for 15 min at 30 °C; flow cytometry was used to detect the differences in the distribution of cell cycles in each group. There was no difference in the proportion of cells in the G1, G2, and S phases among different groups. The results are representative of three independent experiments.

**Figure 8:** Flow cytometry analysis of apoptosis in mimicNC-, mimic584-, inhibitorNC-, and inhibitor584-transfected 16-HBE cells after LPS treatment. The cells were stained with annexin V ± FITC and propidium iodide (PI), and incubated for 15 min in the dark. The fluorescent signal was further analyzed using flow cytometry after the reaction volume was made up to 500 *μ*L by adding a binding buffer. The lower-right panel indicates the percentage of early apoptotic cells (annexin V-stained positive cells). Data are presented as mean ± standard deviation (SD).

**Table 1:** Gene sequences of mimicNC and mimic584.

Name	Sense strand sequence (5′-3′)	Antisense strand sequence (5′-3′)
*Mimic584*	UUAUGGUUUGCCUGGGACUGAG	CAGUCCCAGGCAAACCAUAAUU
*MimicNC(FAM)*	UUGUACUACACAAAAGUACUG	(FAM)GUACUUUUGUGUAGUACAAUU

**Table 2:** Gene sequences of inhibitorNC and inhibitor584.

Name	Sense strand sequence (5′-3′)
Inhibitor584	mCmUmCmAmGmUmCmCmCmAmGmGmCmAmAmAmCmCmAmUmAmA
InhibitorNC	mCmAmGmUmAmCmUmUmUmUmGmUmGmUmAmGmUmAmCmAmA

## Data Availability

The data that support the findings of this study are available from the corresponding author on reasonable request.
